The article "miR-101-3p Contributes to α-Synuclein Aggregation in Neural Cells through the miR-101-3p/SKP1/PLK2 Pathway" was published in 2021. Journal: J Healthc Eng.

# miR-101-3p Contributes to *α*-Synuclein Aggregation in Neural Cells through the miR-101-3p/SKP1/PLK2 Pathway

**DOI:** 10.1155/2021/6147434

**Published:** 2021-06-12

**Authors:** Min Zhang, Wei Liu, Qingan Zhang, Hongfeng Hu

**Affiliations:** Department of Neurology, Jingmen No. 1 People's Hospital, Jingmen, Hubei, China

## Abstract

Parkinson's disease (PD) is a neurodegenerative disorder characterized by progressive neuronal loss in different brain regions, including the dopaminergic (DA) neurons of the substantia nigra pars compacta (SNc). The aggregation of *α*-synuclein (*α*-Syn) plays an essential role in the progression of PD-related neuron toxicity. In this study, bioinformatic analysis was used to confirm differentially expressed genes between patients with PD and healthy donors. Immunofluorescence was used to study the aggregation of *α*-Syn. Flow cytometry was used to confirm the apoptosis of neurons. Western blot was used to investigate the underlying mechanism. Coimmunoprecipitation (co-IP) was used to verify the interaction between proteins. Luciferase activity assay was used to confirm the target gene of miRNA. In vitro protein ubiquitination assay was used to ascertain the role of S-phase kinase-associated protein 1 (SKP1) on the ubiquitination processes of polo-like kinase 2 (PLK2). The result indicated that miR-101-3p was overexpressed in the substantia nigra of the postmortem brains of patients with PD. The underlying role was investigated in the SH-SY5Y cell line. The overexpression of *α*-Syn did not result in toxicity or aggregation. However, the co-overexpression of miR-101-3p and *α*-Syn promoted aggregation and neuron toxicity. Luciferase activity assay indicated that SKP1 is a target gene of miR-101-3p. The co-IP experiment confirmed that SKP1 could directly interact with PLK2. In vitro protein ubiquitination assay confirmed that SKP1 could promote the ubiquitination and subsequent protein degradation of PLK2. We also observed that the cotransfection of short hairpin RNA that targets PLK2 and *α*-Syn overexpression plasmid results in the endoplasmic reticulum stress of neurons. Our results collectively provide evidence that miR-101-3p contributes to *α*-Syn aggregation in neurons through the miR-101-3p/SKP1/PLK2 pathway.

## 1. Introduction

PD is the most common severe movement disorder globally and affects about 1% of adults older than 60 years [1, 2]. The disease is attributed to the selective loss of neurons in the substantia nigra. Its cause is enigmatic in most individuals; PD is characterized by motor and nonmotor symptoms; patients with PD classically display rest tremor, rigidity, bradykinesia, and stooping posture [3–5]. PD can also be associated with neurobehavioral disorders (depression and anxiety), cognitive impairment (dementia), and autonomic dysfunction (e.g., orthostasis and hyperhidrosis) [6, 7]. *α*-Synuclein (*α*-Syn) plays a role in rare familial forms of PD and sporadic PD [8]. Human *α*-Syn is a protein with a molecular mass of ∼14 kDa (containing 140 amino acid residues) and is highly expressed in the brain [8, 9]. The accelerated fibrillation of *α*-Syn may worsen the pathology of PD. Increased *α*-Syn protein levels in the neurons may facilitate its abnormal aggregation, which results in toxicity and diseased condition [10–12].

The article "miR-101-3p Contributes to α-Synuclein Aggregation in Neural Cells through the miR-101-3p/SKP1/PLK2 Pathway" was published in 2021. Journal: J Healthc Eng.

MicroRNAs (miRNAs) are small noncoding RNAs that are transcribed from miRNA genes and intronic sequences as primary miRNAs (pri-miRNAs) and stem-loop precursor miRNAs (pre-miRNAs), respectively [13]. The dysregulation of miRNAs may contribute to the development of various diseases, including brain disorder. Several studies have shown that miRNAs contribute to the progression or onset of PD [14].

A study showed that polo-like kinase 2 (PLK2) expression increased in aged monkeys. PLK2 might play an essential role in the modulation of *α*-Syn [15]. Abid Oueslati et al. reported that PLK2 could interact with *α*-Syn and subsequently promote the autophagic degradation of *α*-Syn [15, 16].

Ubiquitination, which is the process of tagging a protein with ubiquitin, is one of the most versatile cellular regulatory mechanisms [17]. Ubiquitination also participates in multiple cellular processes, including gene transcription and cell cycle progression; ubiquitin degrades protein via the ubiquitin-proteasome system or by selective autophagy [18, 19].

A comprehensive understanding of the association between PD and *α*-Syn is essential to prevent PD progression. In the present study, bioinformatic analysis was used to confirm the differential expression of miR-101-3p in patients with PD and healthy donors. The overexpression of *α*-Syn did not result in toxicity or aggregation, whereas the co-overexpression of miR-101-3p and *α*-Syn promoted aggregation and neuron toxicity. We also found that S-phase kinase-associated protein 1 (SKP1) is a target gene of miR-101-3p and could directly interact with PLK2. We also investigated the underlying mechanisms that contributed to these effects.

## 2. Materials and Methods

### 2.1. Cell Culture and Treatment

Cell line SH-SY5Y cells were purchased from American Type Culture Collection (Manassas, Virginia). The cells were incubated in RPMI-1640 medium (Thermo Fisher Scientific, Inc., Waltham, Massachusetts) supplemented with 10% fetal bovine serum (Gibco, USA) and 100 *μ*g/mL penicillin-streptomycin (Sigma-Aldrich Co, St. Louis, Missouri) and cultured in a humidified atmosphere of 5% CO_2_ in air at 37°C.

The article "miR-101-3p Contributes to α-Synuclein Aggregation in Neural Cells through the miR-101-3p/SKP1/PLK2 Pathway" was published in 2021. Journal: J Healthc Eng.

### 2.2. Transfection

Short hairpin RNAs (shRNAs) for PLK2 and SKP1, overexpression plasmids for PLK2 and *α*-Syn (pcDNA3.1-*α*-Syn), and corresponding negative controls were purchased from Shanghai GenePharma Co., Ltd. (Shanghai, China). miR-101-3p mimic, inhibitor, and negative control were purchased from RiboBio (Guangzhou, China). Transfection was conducted according to the instruction of the manufacturer.

### 2.3. Coimmunoprecipitation (Co-IP)

Cells were lysed with lysis buffer. The lysates were centrifuged and purified by incubation with protein A/G magnetic beads at 4°C for 1 h. The precleared supernatant was then immunoprecipitated with the primary antibody Flag at 4°C overnight. The complexes were subjected to 1 h of incubation at 4°C using protein A/G magnetic beads and subsequently analyzed by Western blot. Of course, we repeated the experiment three times, and the results were recorded.

### 2.4. Western Blot

Western blot was carried out according to the standard protocols described previously. We used primary antibodies against GAPDH (1 : 500; Santa Cruz Biotechnology, CA, USA), *α*-Syn (1 : 1000; #2642), SKP1 (1 : 1000; # 2156S), PLK2 (1 : 1000; # 14812S), eIF2*α* (1 : 1000; #9722), P-eIF2*α* (1 : 1000; #9721), ERK (1 : 500), and P-ERK (1 : 500; Cell Signaling Technology, MA, USA). Goat anti-mouse and anti-rabbit antibodies conjugated with horseradish peroxidase were used as secondary antibodies (1 : 2000; Jackson ImmunoResearch, PA, USA). We detected the blots using enhanced chemiluminescence (Dura, Pierce, NJ, USA). We repeated the experiment three times.

### 2.5. Flow Cytometry

Cell apoptosis was measured by flow cytometry. The cells were harvested and washed with PBS after 24 h of incubation with 1-methyl-4-phenyl-pyridinium (MPP+). Then, the cells were resuspended and incubated with 5 *μ*L of Annexin V-fluorescein isothiocyanate and 5 *μ*L of propidium iodide (PI). Apoptosis percentage, including early apoptosis (Annexin V+/PI−) and late apoptosis (Annexin V+/PI+), was calculated. Experiments were repeated three times to ensure reproducibility. The labeled cells were analyzed using the BD FACSverse flow cytometer (BD, Bioscience), and the data were processed by the FlowJo software (Treestar).

### 2.6. Immunofluorescence Staining

SH-SY5Y cells were fixed with 4% paraformaldehyde for 10 min and permeabilized with PBS containing 0.1% Triton X-100 for 10 min after 72 h of transfection. The cells were blocked in 10% goat serum and incubated overnight with primary antibodies against *α*-Syn (1 : 500; Cell Signaling Technology, MA, USA) at 4°C. The cells were washed with PBS and incubated with fluorescent secondary antibody conjugated with Alexa Fluor®594 for 1 h. Subsequently, the cells were counterstained with 4',6-diamidino-2-phenylindole and imaged with a fluorescence microscope. Fluorescent intensities were measured using the ImageJ software.

The article "miR-101-3p Contributes to α-Synuclein Aggregation in Neural Cells through the miR-101-3p/SKP1/PLK2 Pathway" was published in 2021. Journal: J Healthc Eng.

### 2.7. Statistical Analysis

All statistical analyses in this study were performed using GraphPad Prism 5 for Windows. Data were expressed as mean ± standard deviation (SD) and were compared using a one-way analysis of variance (ANOVA) followed by Tukey's multiple-comparison test. The SPSS 21.0 software was used to analyze the experimental data. A value of *P* < 0.05 was considered statistically significant.

## 3. Results

### 3.1. miR-101-3p and *α*-Syn Co-Overexpression Promotes *α*-Syn Aggregation and Neurotoxicity

Initially, the Gene Expression Omnibus (GEO) database was used to predict the difference in the expression between patients with PD and healthy donors. Figures 1(a) and 1(b) show that the expression of 30 genes considerably changed. Among which, seven genes were upregulated and 24 genes were downregulated in patients with PD. miR-101-3p was the most considerably upregulated among the genes; therefore, miR-101-3p was used in the subsequent study.

The abnormal aggregation of *α*-Syn can promote PD progression and result in neuron toxicity. We confirmed this conclusion by constructing an *α*-Syn overexpression plasmid. The effect of the overexpression was confirmed by Western blot. As shown in Figure 1(c), *α*-Syn was overexpressed successfully. The impact of *α*-Syn overexpression on *α*-Syn aggregation was confirmed by immunofluorescence. Figure 1(c) demonstrates that no remarkable accumulation in SH-SY5Y cells after *α*-Syn was overexpressed. However, the cotransfection of miR-101-3p and *α*-Syn overexpression plasmid resulted in a considerable aggregation of *α*-Syn. Flow cytometry also confirmed that the cell apoptosis rate increased after the co-overexpression of miR-101-3p and *α*-Syn. This finding indicated that the co-overexpression caused substantial neurotoxicity.

Our result indicated that the co-overexpression of miR-101-3p and *α*-Syn promotes *α*-Syn aggregation and neurotoxicity.

### 3.2. miR-101-3p Binds to SKP1 mRNA and Suppresses SKP1 Expression

The public online dataset TargetScan was used to predict the possible target gene of miR-101-3p and confirm the downstream signal pathway of miR-101-3p. We found that SKP1 might serve as the target gene of miR-101-3p. Western blot was performed to confirm this prediction. As shown in Figure 2(a), SKP1 was downregulated after the transfection of miR-101-3p mimic and was upregulated after the transfection of the inhibitor. This result indicated that a regulation relationship might exist between SKP1 and miR-101-3p. Luciferase reporter assay was performed to further confirm their relationship. As shown in Figure 2(b), the 3'-untranslated regions (UTRs) in the predicted binding site of wild-type and mutated SKP1 were constructed, and cDNA was cloned into the luciferase reporter plasmid. The result confirmed that the transfection of miR-101-3p caused a substantial suppression of luciferase activity but did not substantially change the luciferase activity in the luciferase reporter plasmid with mutated UTR. This work demonstrated that miR-101-3p could directly bind to SKP1 mRNA and subsequently suppress SKP1 expression.

The article "miR-101-3p Contributes to α-Synuclein Aggregation in Neural Cells through the miR-101-3p/SKP1/PLK2 Pathway" was published in 2021. Journal: J Healthc Eng.

SKP1 is an essential component of the ubiquitin ligase complex. Therefore, the downstream signal of SKP1 was investigated. As shown in Figure 2(c), the STRING online dataset indicated that SKP1 could interact with PLK2. As shown in Figure 2(d), molecular docking confirmed that PLK2 might directly interact with SKP1. A co-IP experiment was performed based on the evidence.  Figure 2(e) shows that PLK2 precipitated with SKP1; hence, PLK2 could directly interact with SKP1.

Our result confirmed that miR-101-3p targets SKP1 and SKP1 could interact with PLK2.

### 3.3. SKP1 Interacts with PLK2 and Promotes Ubiquitination of PLK2

SKP1 is an essential component of the ubiquitin ligase complex. Therefore, we speculated the interaction between SKP1 and PLK2 might influence the ubiquitination processes of PLK2. To confirm this hypothesis, shRNA targeting SKP1 was constructed, as shown in Figure 3(a); Western blot demonstrated that SKP1 was knocked down successfully, and we select shRNA#3 for subsequent study, as shown in Figure 3(b), after treatment of cycloheximide, a protein synthesis inhibitor, the half-life of PLK1 study. The result confirmed that after downregulation of SKP1, the half-life of PLK2 significantly increased, indicating that downregulation of SKP1 stabilized PLK2 and suppressed the protein degradation processes of PLK2.

To confirm whether SKP1 can influence the ubiquitination processes of PLK2, in vitro protein ubiquitination assay was performed. As shown in Figure 3(c), ubiquitination of PLK2 was enhanced significantly after overexpression of SKP1.

We next investigated the role played by PLK2 in neurotoxicity. To answer this question, PLK2 overexpression vector was constructed, as shown in Figure 3(d); Western blot indicated that PLK2 was overexpressed successfully after transfection of PLK2 overexpression vector.

Neurotoxin MPP+ is a classical neurotoxin that is used to generate a cell model of Parkinson's disease. As shown in Figure 3(e), the apoptosis rate increased after MPP+ treated neuron cells. However, the apoptosis rate was partly reduced after overexpression of PLK2. The result confirmed that PLK2 could partially alleviate neurotoxicity.

The article "miR-101-3p Contributes to α-Synuclein Aggregation in Neural Cells through the miR-101-3p/SKP1/PLK2 Pathway" was published in 2021. Journal: J Healthc Eng.

Our result confirmed that SKP1 interacts with PLK2 and promotes ubiquitination of PLK2, and PLK2 can partly alleviate neurotoxicity.

### 3.4. The Cotransfection of PLK2-Targeting shRNA and *α*-Syn Overexpression Plasmid Promotes Endoplasmic Reticulum (ER) Stress in Nerve Cells

PLK2 can interact with *α*-Syn and subsequently promote the autophagic degradation of *α*-Syn. Co-IP was performed to confirm this conclusion.  Figure 4(a) shows that PLK2 could interact with *α*-Syn. To further investigate the role played by PLK2 in aggregation processes of *α*-syn, shRNA targeting PLK2 was constructed, as shown in Figure 4(b); Western blot indicated that PLK2 was knocked down successfully, and we select shRNA#1 for subsequently study. As shown in Figure 4(c), after cotransfection of PLK2-targeted shRNA and *α*-synuclein overexpression plasmid, P-ERK and eIF2*α* were overexpressed significantly, indicating that cotransfection of PLK2-targeted shRNA and *α*-synuclein overexpression plasmid promotes ER stress.

Flow cytometry was used to confirm our conclusion further. As shown in Figure 4(d), *α*-synuclein overexpression alone does not increase the apoptosis rate. However, cotransfection of PLK2-targeted shRNA and *α*-synuclein overexpression plasmid significantly enhanced apoptosis rate.

Taken together, our result confirmed that cotransfection of PLK2-targeted shRNA and *α*-synuclein overexpression plasmid promotes ER stress in nerve cells.

## 4. Discussion

PD is a severe neurological disease that results from the progressive degeneration of dopaminergic neurons located in the substantia nigra. PD influences about seven million people worldwide and occur among older adults; its prevalence increases from 1% in people aged more than 60 to 4% in those older than 80 [20–22].

MiRNAs with vast regulatory potential have been recently proposed as biomarkers or possible therapeutic targets for PD. MiRNAs are small (about 20–24 nucleotides long), endogenous noncoding RNAs that play a profound role in numerous biological processes in health and disease. Most miRNAs suppress gene expression through the promotion of mRNA degradation and translation inhibition [23]. Previous studies have revealed that miRNAs are implicated in neurodegeneration, and miRNA pathways are affected in almost all neurodegenerative disorders. In this study, the GEO database was used to predict the difference in expression between patients with PD and healthy donors [24]. We found that the expression of 30 genes considerably changed. Among which, seven genes were upregulated and 24 genes were downregulated in patients with PD. miR-101-3p was the most upregulated among the miRNAs. Therefore, miR-101-3p was used for subsequent study [25].

*α*-Syn is a 140-residue natively unfolded protein that is abundantly expressed at the presynaptic terminals. *α*-Syn participates in the regulation of synaptic transmission and dopamine biosynthesis; the overexpression and misfolding of *α*-Syn play an essential role in the progression of neurodegenerative disorders [26, 27]. In the present study, immunofluorescence was used to confirm *α*-Syn aggregation. No remarkable accumulation was observed in SH-SY5Y cells after *α*-Syn was overexpressed [28]. However, the cotransfection of miR-101-3p and *α*-Syn overexpression plasmid resulted in substantial *α*-Syn aggregation. Flow cytometry also confirmed that cell apoptosis rate increased after the co-overexpression of miR-101-3p and *α*-Syn. The results indicated that the co-overexpression caused considerable neurotoxicity.

The article "miR-101-3p Contributes to α-Synuclein Aggregation in Neural Cells through the miR-101-3p/SKP1/PLK2 Pathway" was published in 2021. Journal: J Healthc Eng.

SKP1 is an essential component of the ubiquitin ligase complex. In this study, we confirmed that SKP1 can bind to PLK2 and subsequently promote the ubiquitination of PLK2.

PLK2 can bind directly to *α*-Syn and regulate *α*-Syn clearance [29–31]. In the current study, we confirmed that *α*-Syn could directly interact with PLK2, and the overexpression of PLK2 can partly alleviate the neurotoxicity induced by MPP+. The binding between PLK2 and *α*-Syn is needed for *α*-Syn clearance.

Based on our result, miR-101-3p overexpression in neurons may suppress the expression of SKP1. SKP1 downregulation limited the clearance of *α*-Syn and subsequently caused the abnormal accumulation and aggregation of *α*-Syn.

Our result provides evidence that miR-101-3p contributes to *α*-Syn aggregation in neurons through the miR-101-3p/SKP1/PLK2 pathway.

## Figures and Tables

**Figure 1:** Co-overexpression of miR-101-3p and *α*-synuclein promotes *α*-Syn aggregation and neurotoxicity. (a) Heatmap of gene expression between substantia nigra from postmortem brains of patients with Parkinson's disease and health donors. (b) Volcano map of gene expression between substantia nigra from postmortem brains of patients with Parkinson's disease and health donors. (c) Western blot analysis of SH-SY5Y after transfection of *α*-synuclein overexpression plasmid. (d) Immunofluorescence of *α*-synuclein aggregation. (e) Flow cytometry analysis of cell apoptosis. Error bars represent mean ± SD. ^*∗∗*^*P* < 0.01. n.s., not significant, by the paired two-sided Student's *t*-test.

The article "miR-101-3p Contributes to α-Synuclein Aggregation in Neural Cells through the miR-101-3p/SKP1/PLK2 Pathway" was published in 2021. Journal: J Healthc Eng.

**Figure 2:** miR-101-3p binds to mRNA of SKP1 and suppress SKP1 expression. (a) Western blot analysis of SKP1 expression in SH-SY5Y after transfection of miR-101-3p mimic or inhibitor. (b) Illustration of SKP1 3'UTR and SKP1 3' UTR mutation. Right panel, quantification of the luciferase activity. (c) Protein-protein interaction predicted by the STRING online dataset. (d) Molecular docking of PLK2 and SKP1. (e) Co-IP experiment of SKP1 and PLK2. Error bars represent mean ± SD. ^*∗∗*^*P* < 0.01. n.s., not significant, by the paired two-sided Student's *t*-test.

**Figure 3:** SKP1 interact with PLK2 and promotes ubiquitination of PLK2. (a) SKP1 expression after SH-SY5Y was transfected by shRNA targeting SKP1. (b) Half-life of PLK2 evaluated after treated by cycloheximide. (c) Ubiquitination assay of PLK2 with or without SKP1 overexpression. (d) Western blot analysis of PLK2 after transfection of PLK2 overexpression plasmid. (e) Flow cytometry analysis of cell apoptosis.

**Figure 4:** Cotransfection of PLK2-targeted shRNA and *α*-synuclein overexpression plasmid promotes ER stress in nerve cells. (a) Co-IP experiment of PLK2 and *α*-synuclein. (b) Western blot analysis of PLK2 after transfection of shRNA targeting PLK2. (c) Western analysis of P-ERK and P-eIF2*α*. (d) Flow cytometry analysis of cell apoptosis. Error bars represent mean ± SD. ^*∗∗*^*P* < 0.01. n.s., not significant, by the paired two-sided Student's *t*-test.

## Data Availability

The data used to support the findings of this study are available from the corresponding author upon request.
